# Cytokinins: A Genetic Target for Increasing Yield Potential in the CRISPR Era

This article has been retracted.

**DOI:** 10.3389/fgene.2022.883930

**Published:** 2022-04-26

**Authors:** Sayanti Mandal, Mimosa Ghorai, Uttpal Anand, Debleena Roy, Nishi Kant, Tulika Mishra, Abhijit Bhagwan Mane, Niraj Kumar Jha, Milan Kumar Lal, Rahul Kumar Tiwari, Manoj Kumar, Radha, Arabinda Ghosh, Rahul Bhattacharjee, Jarosław Proćków, Abhijit Dey

**Affiliations:** ^1^ Institute of Bioinformatics and Biotechnology, Savitribai Phule Pune University, Pune, India; ^2^ Department of Life Sciences, Presidency University, Kolkata, India; ^3^ CytoGene Research & Development LLP, Barabanki, Uttar Pradesh, India; ^4^ PG Department of Botany, Lady Brabourne College, Kolkata, India; ^5^ Department of Biotechnology, ARKA Jain University, Jamshedpur, India; ^6^ Department of Botany, DDU Gorakhpur University, Gorakhpur, India; ^7^ Department of Zoology, Dr. Patangrao Kadam Mahavidhyalaya, Ramanandnagar (Burli), Sangli, India; ^8^ Department of Biotechnology, School of Engineering and Technology, Sharda University, Greater Noida, India; ^9^ ICAR-Central Potato Research Institute, Shimla, India; ^10^ Chemical and Biochemical Processing Division, ICAR-Central Institute for Research on Cotton Technology, Mumbai, India; ^11^ School of Biological and Environmental Sciences, Shoolini University of Biotechnology and Management Sciences, Solan, India; ^12^ Microbiology Division, Department of Botany, Gauhati University, Guwahati, India; ^13^ School of Biotechnology, Kalinga Institute of Industrial Technology (KIIT) Deemed To Be University, Bhubaneswar, India; ^14^ Department of Plant Biology, Institute of Environmental Biology, Wrocław University of Environmental and Life Sciences, Wrocław, Poland

**Keywords:** cytokinin, cytokinin oxidase/dehydrogenase, IPT, CRiSPR/Cas, crop improvement

## Abstract

Over the last decade, remarkable progress has been made in our understanding the phytohormones, cytokinin’s (CKs) biosynthesis, perception, and signalling pathways. Additionally, it became apparent that interfering with any of these steps has a significant effect on all stages of plant growth and development. As a result of their complex regulatory and cross-talk interactions with other hormones and signalling networks, they influence and control a wide range of biological activities, from cellular to organismal levels. In agriculture, CKs are extensively used for yield improvement and management because of their wide-ranging effects on plant growth, development and physiology. One of the primary targets in this regard is cytokinin oxidase/dehydrogenase (CKO/CKX), which is encoded by CKX gene, which catalyses the irreversible degradation of cytokinin. The previous studies on various agronomically important crops indicated that plant breeders have targeted CKX directly. In recent years, prokaryotic clustered regularly interspaced short palindromic repeats (CRISPR)/CRISPR-associated protein 9 (Cas9) system has been increasingly used in editing the CKO/CKX gene and phenomenal results have been achieved. This review provides an updated information on the applications of CRISPR-based gene-editing tools in manipulating cytokinin metabolism at the genetic level for yield improvement. Furthermore, we summarized the current developments of RNP-mediated DNA/transgene-free genomic editing of plants which would broaden the application of this technology. The current review will advance our understanding of cytokinins and their role in sustainably increase crop production through CRISPR/Cas genome editing tool.

## Introduction

As a result of climate change and decreasing biodiversity, recent efforts in crop breeding programmes have focused on increasing tolerance to disease and environmental stress (Bellard et al., 2012; Mills et al., 2018). Furthermore, little progress is being made in terms of increasing the yield potential and agricultural productivity (Fugile, 2018). One of the most significant consequences of a growing global population is the need to provide ever-increasing amounts of food, fibre, and fuel while also acknowledging the need for sustainable production methods that operate in a changing global environment. In order to meet this growing requirement, the seed production is critical as it provides the raw material for fibre, fuel and food (Raza et al., 2019). Moreover, it has been noted that there is frequently a conflict between the seed production and the final end-product (food). Seed yield optimization must be done while maintaining the quality of the fibre, fuel, or food (vegetable, forage, cereal).

Cytokinins have been linked to seed development as high levels were detected during the process of seed development which led to the discovery of the first naturally occurring cytokinin, zeatin, from *Zea mays* (Letham, 1963) (Figure 1). It is possible to use modern biotechnology tools along with the traditional breeding for crop improvement. With the invent of new biotechnological tools (NBTs), such as marker-assisted selection (MAS), next-generation sequencing (NGS), genome editing (GE), and genetic transformation protocols, can be used as an additional tool along with the traditional breeding methods.

**FIGURE 1:** Various natural and synthetic cytokinins (structures obtained from www.ChemSpider.com) **(A)** kinetin, **(B)** zeatin, **(C)** 6-benzylaminopurine, **(D)** Diphenylurea, **(E)** thidiazuron (TDZ).

In these efforts, novel GE tools could be particularly useful. In the field of GE, CRISPR/Cas (clustered regularly interspaced short palindromic repeat/CRISPR associated Cas) is considered a breakthrough technology, primarily due to its high efficacy and ease of implementation. As a foundation, CRISPR/Cas technology allows for the introduction of precise knockout mutations at specific genomic locations. Additionally, this system can be used to introduce defined mutations (gene repair), stack genes, or regulate gene expression in more advanced approaches (Bortesi and Fischer, 2015; Nidhi et al., 2021). Moreover, large number of crops are successfully edited through CRISPR/Cas tool because of its precision, simplicity and relatively cheaper (Jaganathan et al., 2018). Furthermore, induced mutations were found to be stably inherited in progeny plants. Additionally, with the availability of genome sequences for many crops and efficient genetic transformation protocols in recent years, various advanced forms of CRISPR have become readily available for use (Hensel et al., 2009; Mascher et al., 2017). Increased crop productivity is one of the major goals in agriculture, alongside adaptation to various biotic and abiotic stress. Manipulation of cytokinin (CK) metabolism is a promising tool for increasing plant productivity.

A wide range of physiological processes are regulated by the naturally occurring cytokinins, that stimulate cell division, root formation and regulate shoot, and are involved in the growth and development of leaves, flowers and fruits (Kieber and Schaller, 2018; Vankova, 2014). The regulators of cytokinin metabolism and signalling are particularly interesting among these genes because the effects of cytokinin activity on seed development is well established (Jameson and Song, 2016). Cytokinins are a sign of high physiological activity, and as a result, plants have evolved a variety of mechanisms to regulate the levels of active cytokinin at different developmental stages. Members of several multigene families are responsible for cytokinin biosynthesis (isopentenyl transferase, IPT), activation (LONELY GUY, LOG), irreversible degradation (cytokinin oxidase/dehydrogenase, CKX), reversible inactivation (zeatin O-glucosyltransferase, ZOG), and reactivation (glucosidase, GLU). Cytokinin oxidase/dehydrogenase enzymes (CKX) catalyse the degradation of cytokinin by cleaving the active cytokinin form’s unsaturated isoprenoid side chains. A family of CKX genes encodes CKX enzymes with tissue specificity and developmentally dependent expression patterns (Werner et al., 2006). The CKX genes, which are important regulators of cytokinin levels, have attracted the attention of researchers, who have noted their potential for crop improvement as a result of their ability to manipulate cytokinin homeostasis in plants. Evidently, several studies have demonstrated that suppressing the expression of CKX can improve the quality of some crop yield attributes in some cases. In rice, barley, cotton, and Arabidopsis, for example, downregulation of CKX genes via mutation, RNAi-based silencing, or genome editing (CRISPR) resulted in higher seed numbers and/or seed weight (Bartrina et al., 2011; Zalewski et al., 2012; Li et al., 2013; Zhao et al., 2015; Li et al., 2016). Additionally, it has been demonstrated that CKX genes have an effect on root growth and morphology (Werner et al., 2003; Mrízová et al., 2013).

Alternatively, homeostasis of cytokinins can be manipulated by overexpression of IPT genes. IPT is a member of a small family of genes that encode isopentenyl transferases, which are directly involved in the *de novo* synthesis of cytokinin hormones. In barley, IPT genes, like CKXs, indicate tissue specificity and development-dependent expression patterns (Mrízová et al., 2013). Numerous crop plants have benefited from ectopic IPT gene expression during seed production (Jameson and Song, 2016). This review provides an overview of molecular aspect of cytokinin actions that regulates various physiological process in the plant. Furthermore, we also highlight the current progress on the applications of CRISPR/Cas9 and various other molecular technique in increasing grain yields by manipulated the CKX gene. Finally, we also discussed the CRISPR/Cas9 DNA-free editing in crops that has a great prospect of being commercialized.

## Molecular Basis of Cytokinin Regulation

Physiological and developmental processes include apical dominance release, axillary shoot branching, root meristem cell patterning, and the formation of lateral roots, are controlled by CKs in plants through a complex network of cross-talk between signaling pathways (Koprna et al., 2016). In addition to playing a critical role in the regulation of plant cell proliferation and differentiation, they are involved in the regulation of a variety of processes in plant growth and development. These include the inhibition of root development, the promotion of shoot growth, development of seed and fruit, delaying of the onset of senescence, the transduction of nutritional signals, and the response to both biotic and abiotic stresses (Koprna et al., 2016; Cortleven et al., 2019). To maintain cytokinin homeostasis and regulate a variety of physiological processes, bioactive molecules are synthesised, activated, degraded, and conjugated (Figure 2).

**FIGURE 2:** Schematic representation for the cytokinin biosynthesis and degradation pathways.

Cytokinins are produced by nearly every living organism. Cytokinins are naturally occurring adenine derivatives with isoprenoid or aromatic side chains at the adenine ring’s N6 position (Kiba et al., 2013). Thus, natural cytokinins can be classified into isoprenoid and aromatic CKs, with the former being more abundant in plants (Sakakibara, 2006). The most important components of isoprenoid cytokinins are trans-zeatin (tZ), isopentenyl adenine (iP) and cis-zeatin (cZ), with iP and tZ being the most active (Sakakibara, 2006; Kudo et al., 2010). The aromatic cytokinins entail orthotopolin (oT), mesotopolin (mT), their methoxy derivatives (MemT and MeoT), benzyladenine (BA), and more. These, on the other hand, are found only in a few plant species, such as *Nicotiana tabacum* and poplar (Sakakibara, 2006; Kudo et al., 2010). The terpenoid pathway is responsible for the synthesis of cytokinin. The enzymes LONELY GUY (LOG) and isopentenyl transferase (IPT) are two of the most important players in cytokinin biosynthesis (Kuroha et al., 2009). Adenosine phosphate-isopentenyl transferases and tRNA-isopentenyl transferases (tRNA-IPTs) make up the majority of IPTs, which serve as the primary rate-limiting enzymes in cytokinin biosynthesis. The IPPT-binding domain of these two types of IPTs is conserved, which is a characteristic shared by both the enzymes (Sakakibara, 2006). The adenosine phosphate-isopentenyl transferases can catalyze dimethylallyl diphosphate (DMAPP) to form iP-ribotides, which are precursors of iP that initiates cytokinin biosynthesis (Sakakibara, 2006; Kudo et al., 2010). The cytochrome P450 monooxygenase CYP735As catalyses the conversion of iP-ribotides to tZ-ribotides, which is also important in promoting shoot growth of *Arabidopsis thaliana* (Kiba et al., 20013). Furthermore, iP- and tZ-ribotides are the precursors of the majority of iP- and tZ-type cytokinins (Kudo et al., 2010).

The synthesis of cZ starts with tRNA-IPTs, which use DMAPP to help with the prenylation of tRNA and then generats cZ-ribotides (Sakakibara, 2006). In some plants, multiple gene families encode IPTs; for example, *A. thaliana* has 9 IPTs (*AtIPT1*-*AtIPT9*), *Oryza sativa* has 10 IPTs (*OsIPT1*-*OsIPT10*), and the *Fragaria × ananassa* has 7 *FvIPTs* (Frebort et al., 2011; Zurcher and Muller, 2016). The lysine decarboxylase-binding domain of all the proteins expressed by LOGs which is conserved across the plant kingdom and a new discovered cytokinin-activating enzyme (Mi et al., 2017). In the next step, LOGs convert inactive cytokinin ribotides into biologically active free base form through their cytokinin-specific phosphohydrolase activity (Kudo et al., 2010). The first LOGs were discovered in *O. sativa*, and the nine LOGs (*AtLOG1*-*AtLOG9*) discovered in *A. thaliana* were later thought to be rice homologs (Kuroha et al., 2009). The *Fragaria × ananassa* genome recently revealed the presence of nine *FvLOGs*. Under osmotic stress, high temperature treatment, and exogenous abscisic acid (ABA), the expression of most *FvLOGs* and *FvIPTs* changes, suggesting that these genes may play a role in plant resistance to abiotic stresses (Mi et al., 2017).

Plants require precise control of biosynthesis and metabolic enzymes to maintain cytokinin levels. Biosynthesis and metabolic enzymes must be tightly regulated in plants in order to maintain cytokinin levels and regulate numerous physiological and biochemical process. As a result, not only cytokinin synthetase, but also cytokinin-metabolizing enzymes are required to maintain stable cytokinin levels (Frebort et al., 2011). The level of active cytokinin can be controlled by binding to sugars (mostly glucose) or by irreversible cleavage of cytokinin oxidases, which are enzymes that degrade active cytokinin (CKXs) (Werner et al., 2006). Glucose binds to cytokinin at the purine ring’s N3, N7, and N9 positions or the hydroxyl group of the pentenyl side chain, including O and N-glycosylation (Kudo et al., 2010). Glucosyltransferase catalyses O-glycosylation on the oxygen of the cytokinin side chain, which is reversed by β-glucosidase (Sakakibara, 2006). Purine ring N-glycosylation, which mainly occurs on the N7 or N9 purine ring, is considered to be irreversible (Sakakibara, 2006; Kudo et al., 2010). In bioassays, glucosyl conjugates are inactive, and the bounded cytokinins are unable to bind to histidine kinase (HK) cytokinin receptors (Spichal et al., 2004). It has been demonstrated that cytokinins bound to glucosyl conjugates do not bind to the receptors for histidine-kinase (HK) cytokinins in biological assays. CKXs are the only enzymes known to catalyse the irreversible degradation of cytokinin (Galuszka et al., 2007; Kudo et al., 2010). Flavin adenine dinucleotide (FAD) binding and substrate binding are two conserved domains in mature CKXs that have different biochemical functions and subcellular localization (Galuszka et al., 2007; Kowalska et al., 2010). By irreversibly cutting the free radicals and ribose forms of cytokinins on the N6 side chain, CKXs lower the level of active cytokinins (Werner et al., 2006). CKXs cleave both tZ and iP, but DZ, synthetic cytokinin kinetin, and 6-benzylaminopurine are resistant to cleavage (Galuszka et al., 2007). Furthermore, manipulating CKXs has a significant impact on endogenous cytokinin levels, which is discussed in great detail in the following section.

## Role of Cytokinin in Improving Crop Yield

Cytokinin oxidases/dehydrogenases (CKX) are involved in the regulation of cytokinin-dependent processes and are important in controlling endogenous cytokinin levels (Schmüllin et al., 2003). CKX is considered to act as a negative regulator of cytokinin production and may be involved in grain development (Galuszka et al., 2001). In the early stages of grain development in *Oryza sativa* (rice), cytokinin plays an important role in regulating grain filling pattern, which in turn affects grain filling percentage. Moreover, it is evident in rice endosperm, cell division is regulated by CK in the grains at the early stages of grain development (Yang et al., 2000; Yang et al., 2003). Furthermore, stay-green traits and senescence are closely linked through CK, which acts as a general coordinator between the two. *Triticum aestivum* (wheat) yields can be increased by using stay-green, as well as its resistance to heat stress during active photosynthesis (Yang et al., 2016). The improvement of leaf anatomical and biochemical traits, including tolerance to suboptimal temperature conditions, can lead to high yields by increasing photosynthetic productivity (Brestic et al., 2018). Numerous scientific studies indicate that the overexpression of the CKX gene resulted in a decrease in the endogenous cytokinin content of plants (Jones and Schreiber, 1997). The role of CKX in many agronomically important crops was elucidated using transgenic and genome-editing technology, which is discussed in detail in the following section. Table 1 summarises the genetic and molecular approaches applied for manipulating the cytokinin gene in a variety of crop plant.

**TABLE 1:** Summary of cytokinin oxidase/dehydrogenase (CKX) expression/activity on yield attributes in agronomically important crops.

S. No	Cultivar	Technique used	Gene	Observation	Reference
*Oryza sativa* (Cereal)					
1	*O. sativa* ssp. *japonica* cv. Nipponbare and Zhonghua 11	CRISPR/Cas9	*OsCKX4* and *OsCKX9*	The double mutant had a significantly greater number of tillers, compared to the wild type	Rong et al. (2021)
2	*O. sativa* ssp. *japonica* cv. Nipponbare	CRISPR/Cas9	*OsCKX11*	Genome edit lines were found to be effective in delaying leaf senescence, increasing grain number, and coordinating source and sink regulation	Zhang et al. (2021)
3	*O. sativa* ssp. *japonica* cv. Nipponbare and Wuyunjing 30	Overexpression lines	*RGG1*	Cytokinin content was found to be lower in the overexpression lines	Tao et al. (2020)
4	*O. sativa* cv. Nipponbare	RNAi and CRISPR/Cas9	*OsNAC2* (encodes a NAC TF)	The primary root length and number of crown roots both were increased in the modified plant	Mao et al. (2019)
5	*O. sativa* cv. Nipponbare	Overexpression lines	*Os6*	Identified in rice that glycosylated cytokinin *in vitro*	Li et al. (2019)
6	*O. sativa* ssp. *japonica* cv. Nipponbare and Zhonghua 11	CRISPR/Cas9, overexpression lines	*CKX9* (responds only to strigolactone)	Mutants and overexpressing transgenic plants both exhibited significant increases in tiller number while simultaneously experiencing significant decreases in panicle size and plant height	Duan et al. 2019
7	*O. sativa* cv. Zhonghua 11	Overexpression lines	*OsAFB6* (*Auxin-signaling F-Box 6*)	Transgenics lines significantly increased the number of spikelets per panicle and primary branch number all led to a 50% increase in grain yield	He et al. (2018)
8	*O. sativa* cv. TNG67	RNAi	*OsCKX2*	Transgenic crop demonstrated improved yield with increased tiller number	Yeh et al. (2015)
9	*O. sativa* cv. Koshihikari	RNAi and overexpressed lines	*OsCKX2* (*Gn1a*)	The number of reproductive organs in transgenic lines increased, resulting in increased grain yield	Ashikari et al. (2005)
*Triticum aestivum* (Cereal)					
10	*T. aestivum* cv. Paragon and Bobwhite	CRISPR/Cas9 and TILLING	*GW2*	Increased GS and TGW were observed in the knockout mutant	Wang et al. (2018)
11	*T. aestivum* cv. Kenong 9204	RNAi	*Ta2.2.1-3A*	Displayed increased grain yield	Li et al. (2018)
12	*T. aestivum* cv. Kontesa	RNAi	*TaCKX1*	Transgenic lines had a positive effect on plant productivity	Zalewski et al. (2010)
*Hordeum vulgare* (Cereal)					
13	*H. vulgare*	CRISPR/Cas9	*HvCKX1*, *HvCKX3*	The root phenotype of the knockout mutant was altered, but grain yields were not increased	Gasparis et al. (2019)
14	*H. vulgare* cv. Golden Promise	RNAi and CRISPR/Cas9	*HvCKX1*	Transgenic lines exhibited decreased root growth, but they had more tillers and grains than WT, and the total yield increased to 15%	Holubová et al. (2018)
15	*H. vulgare* cv. Golden Promise	Transgenic lines	*AtCKX1*, *AtCKX2*	Transgenic plants have larger root systems and are able to withstand long-term droughts than WT.	Ramireddy et al. (2018)
16	*H. vulgare* cv. Golden Promise	Transgenic lines	*AtCKX1*	Roots with higher drought tolerance were observed in the overexpressing line	Pospíšilová et al. (2016)
17	*H. vulgare* cv. Golden Promise	Overexpression lines	*HvCKX1*	Overexpression plant lines were unable to flower with rapid root proliferation and high root-to-shoot ratios	Mrizová et al. (2013)
18	*H. vulgare* cultivar Golden Promise	RNAi	*HvCKX1*, *HvCKX2*	Transgenic lines resulted in increased productivity which was achieved through increased seed production and grain yield	Zalewski et al., 2010; 2012
*Jatropha curcas* (Biofuel)					
19	*J. curcas*	CRISPR/Cas9	*IPTs*, *CYP735A* and *CKXs*	Displayed spatio-temporal expression	Cai et al. (2018)
*Brassica napus* (Oilseed)					
20	*B. napus* cv. Kristina	Transgenic plants	*AtCKX2*	The transgenic lines developed displayed increased number of lateral and adventitious roots. Moreover, the leaves of transgenic plants accumulated higher levels of macro- and microelements	Nehnevajova et al. (2019)
*Solanum tuberosum* (Tuber crop)					
21	*S. tuberosum* cv. Désirée	Overexpression lines	*AtCKX2*	Overexpressing lines exhibited fewer shoot and remarkably increased CKX activity. Under inducing conditions, tuberization was found to be improved in these lines	Raspor et al. (2012)

Abbreviations: RNAi, RNA interference; TF, transcription factor; GS, grain size; TGW, thousand grain weight.

Earlier published reports in 2001, demonstrated that overexpression of the *AtCKX* gene in *N. tabacum* plants resulted in decreased endogenous cytokinin levels (Werner et al., 2001). Zeng et al. (2012) found that the *Gossypium hirsutum* L. gene *GhCKX* was suppression or overexpression in the model plant *N. tabacum*, resulting in over-production of cytokinin (e.g., more capsules and flowers) or deficiency of cytokinin (e.g., fewer or no flowers). Another group of researchers identified that bigger roots, smaller shoots, and smaller shoot apical meristems (SAMs) in *A. thaliana* when *AtCKX1* and *AtCKX2* genes were overexpressed. But overexpression of *AtCKX7* in the model plant results shorter primary roots were reported (Kollmer et al., 2014; Werner et al., 2001). In addition, *ckx3 ckx5* double mutants had more siliques and larger SAM (Bartrina et al., 2011). The findings support the critical role of cytokinin in a variety of model plants.

Zalewski et al. (2010) used hairpin RNA interference to successfully silenced the expression of *HvCKX1* and *TaCKX1* gene resulting in lower CKX activity and significant increase in grain productivity and greater root weight in *Hordeum vulgare*. Raspor et al. (2012) and team overexpressed the *AtCKX2* gene in *Solanum tuberosum* L. cv. Désirée that resulted in significantly lower levels of bioactive cytokinins when compared to the control. Furthermore, Mrìzová et al. (2013) found that overexpression of CKX induces CK-deficiency in *H. vulgare*, prevents them from flowering and resulting morphological changes such as distinctively enlarged root systems and retarded development of aerial parts. The overexpressed plants also displayed higher root-to-shoot ratios when compared to wild-type (WT). Gu et al. (2015) utilized the *An-2* gene (from *Oryza sativa*) encoding for Lonely Guy like protein 6, was cloned into *O. rufipogon* (brownbeard rice) exhibited a pleiotropic effect on root length, tiller number, grain number and awn length. Cloned *An-2* in the *O. rufipogon* background increased the endogenous cytokinin concentration, which promoter rice awn elongation. In a different study, use of RNAi mediated silencing of rice cytokinin gene showed downregulation of *OsCKX2* that led to a higher tiller number and grains per with delayed senescence (Yeh et al., 2015). He et al. (2018) overexpressed the *OsAFB6* (*Auxin-signaling F-Box 6*) which increased the cytokinin levels by supressed the *Gn1a* (*OsCKX2*) and increase the IAA concentration in the rice panicle. In the overexpressed lines, the increased cytokinin delayed heading but improved grain yield. In *Jatropha curcas*, CRISPR/Cas9 technology was used to create knockout mutants of *JcCYP735a*, which resulted in significantly lower concentrations of tZ and tZ-riboside (tZR), as well as severely stunted growth (Cai et al., 2018). In addition, Halubavaet et al. (2018) generated CRISPR mediated knock out of *HvCKX1* gene generated homozygous transgenic plants with reduce root growth and increase in grain productivity. Li et al. (2018) focused on silencing the *TaCKX2.4* gene in *Triticum aestivum*, which reduced the activity of the cytokinin oxidase in transgenic plants, resulting in cytokinin accumulation. Increased cytokinin accumulation in inflorescence meristems results in an increase in the number of reproductive organs, which leads to an increase in the number of grains per spike, spike length, thousand-grain weight (TGW), seed length, and seed width. In *H. vulgare*, Gasporis et al. (2019) reported CRISPR-mediated knockout of the *HvCKX1* and *HvCKX3* genes. The CKX enzyme was found to be lower in the spikes of these knockout, and the root surface, morphology, and hair were all greater in comparison to the WT. Increased cytokinin glycoside levels were observed in *A. thaliana* overexpressing the rice Os6 cytokinin glycosyltransferase gene (Li et al., 2019). In addition, Nehnevajova et al. (2019) found that overexpressing the *AtCKS2* gene in oilseed *Brassica napus* increased the root-to-shoot ratio. CRISPR-edited RGG1 (G proteins) in *O. sativa* decreased endogenous cytokinin levels and reduced grain size and plant development, as demonstrated by Tao et al. (2020). It has been shown that during leaf senescence *OsCKX11* plays an antagonistic role in both the cytokinin and abscisic acid (ABA) pathways. The downregulation of ABA biosynthesis genes and the upregulation of ABA degradation genes in CRISPR/Cas9 edited *osckx11* mutants result in a reduction of ABA content in flag leaves and, as a result, regulate leaf senescence, demonstrating the relationship between cytokinin and ABA. These results show that *OsCKX* genes serve as a link between cytokinin and other plant hormones (Zhang et al., 2021). Similarly, in 2021, Rong et al. demonstrated an efficient method of CRISPR-mediated genome editing in rice cultivars Nipponbare and Zhonghua 11 to create knock out mutants of *OsCKX4* and *OsCKX9* gene. The mutant had a higher number of tillers than the wild type in both field and pot experiments. In comparison to the control, the double mutant *osckx 4* and *osckx 9* created through genome editing techniques had a higher tiller number. These findings shed light on the functions of *CKX* genes in a variety of crop species and could serve as a foundation for future research aimed at increasing yield potential.

## CRISPR/Cas9: A Rapidly Evolving Biological Tool for Editing Plant Cytokinin

### CRISPR/Cas9: Mechanism

The Clustered regularly interspaced short palindromic repeats/CRISPR-associated nuclease9 (CRISPR/Cas9) gene editing system was designed on the adaptive immune defence mechanism that the bacteria used to attack the entering viruses and plasmids (Pramanik et al., 2020). In a nutshell, CRISPR/Cas-mediated editing works by using short RNA sequences called guide RNAs (gRNAs) to complementarily target DNA, which is then cleaved by a Cas endonuclease. The DNA cleavage recognition motif, known as a protospacer adjacent motif (PAM), is found on the endonuclease. A few base pairs away from the PAM, the Cas protein cleaves DNA. CRISPR/Cas, like other methods of gene editing, takes advantage of two different types of DNA repair mechanisms i.e., nonhomologous end-joining (NHEJ) and homologous recombination (HR). In plant cells, NHEJ is the primary repair mechanism, and its imprecise repair results in indels (insertions or deletions) within a gene sequence, causing gene expression to be disrupted (Puchta, 2005). The knockout lines generated are often used in reverse genetics to decipher the role and function of a particular genes. But at the other hand, plant cells are less likely to repair themselves through HR because it is much less effective than NHEJ (Schmidt et al., 2019). Additionally, homology-directed repair (HDR) is a technique that involves delivering a DNA repair template along with the CRISPR/Cas components in order to insert a DNA sequence. Moreover, HDR is inefficient in plants, with only one in every 10^5^–10^4^ transformation events, owing primarily to the fact that NHEJ is the principal repair mechanism in plants (Horvath and Barrangou 2010).

### CRISPR/Cas9: Development of the Genome Editing Tools

Discovered in 1987 by Japanese scientists, the *Escherichia coli* genome contained some previously unknown tandem repeats, but they did not investigate further for their biological role (Ishino et al., 1987). Although these sequences were given the name Clustered Regularly Interspaced Short Palindromic Repeats (CRISPR) in 2002, the significance of these sequences remained unknown until recently (Jansen et al., 2002). Protospacer-adjacent motifs (PAMs) were discovered by three separate research groups in 2005, and it was hypothesised that they would guide the type II Cas9 nuclease to cut DNA (Mojica et al., 2005; Bolotin et al., 2005). Barrangou et al., in 2007, established that the CRISPR system is indeed a prokaryotic adaptive immune system, demonstrating that bacteria can change their resistance to phages by incorporating phage gene sequences (Barrangou et al., 2007). Brouns et al., in 2008 discovered that in order to perform a defensive action, the non-coding RNA transcribed from the CRISPR proto-inter-regional sequence guides the Cas protein to target-specific part of DNA (Brouns et al., 2008). Deltcheva et al. demonstrated in 2011 that trans-coding crRNA (tracrRNA) is involved in the pre-crRNA processing and maturation process, and their research identified new pathways for crRNA maturation (Deltcheva et al., 2011). Furthermore, *in vitro* experiments in 2012 showed that mature crRNA formed a unique double-stranded RNA structure with tracrRNA through base complementary pairing, directing Cas9 protein to cause double-stranded DNA break (Jinek et al., 2012). It has been well established that the CRISPR/Cas9 system has successfully edited numerous agronomical traits in an variety of crop species (Jaganathan et al., 2018). Additionally, the dCas9 protein mutant (endonuclease-deficient) was first created in 2013, losing its nuclease activity (Qi et al., 2013). By fusing the dCas9 protein with transcription regulators that activate or inhibit gene transcription, the CRISPR activation (CRISPRa) and interference (CRISPRi) tools were developed (Figure 3) (Maeder et al., 2013; Gilbert et al., 2013). To address the issue of unexpected disruptions in the CRISPR/Cas9 gene editing system, Komor et al. fused APOBEC (cytosine deaminase) with CRISPR/Cas9. Under the guidance of gRNA, this modified Cas9 performs the C→T (or G→A) conversion without causing DSB. With the help of this base editor, a variety of point mutations in the genome could be successfully corrected (Komor et al., 2016). In addition, the Adenine Bases Editor (ABE) was created to convert A-T base pairs to G-C base pairs (Figure 3) (Gaudelli et al., 2017). The single-base editing and CRISPR/Cas9 systems were further improved by the team, which resulted in a significant decrease in the miss rate of the single-base editor and an increase in the target range of spCas9, respectively (Doman et al., 2020; Miller et al., 2020). Gilpatrick et al., for instance, used Cas9 and adapter ligation to develop a nanopore Cas9-targeted sequence (nCATS) for third-generation nanopore sequencing by modifying the target DNA region and altering the target genome’s structure, allowing for the reading of long fragments at a low cost (Gilpatrick et al., 2020). Recently, researchers developed a caged RNA strategy that enables Cas9 to bind to DNA but does not cleave prior to light-induced activation. This method was known as very fast CRISPR (vfCRISPR) that creates double-strand breaks (DSBs) at the submicrometer and second scales (Figure 3). Due to the high accuracy of the vfCRISPR and the ability to edit only one allele at a time, it can be used to investigate complex genetic traits (Lino et al., 2018). Taken together, these advancements enabled the CRISPR/Cas9 transition from a blunt to a precise genome editing tool.

**FIGURE 3:** Proposed CRISPR/Cas9 applications to target cytokinin in crop plants. CRISPR knock out (CRISPR KO) is presently successfully applied (reported in the review). We propose CRISPR-Base-Editing and Prime-Editing, CRISPRi, CRISPRa and vfCRISPR can also be used in this regard.

### CRISPR/Cas9: RNP-Mediated DNA-Free Genome Editing

Plant cells and tissues are most commonly targeted by Agrobacterium or particle bombardment-mediated transformation with DNA containing CRISPR expression cassettes. This is the most common method for the delivery of CRISPR reagents, such as Cas proteins and gRNAs, into plants. Concerns and regulatory burdens arise from the random integration of CRISPR cassettes into plant genomes. There are concerns about the random integration of CRISPR cassettes into genomes which results in imposing regulatory burden. Breeding can be used to remove these transgene elements, but this process is time- and labor-intensive, making it unsuitable for species or varieties that have long juvenile growth periods or that are typically vegetatively propagated, making it impractical. It has been possible to generate transgene-free genome-edited plants by using transient expression of transgenes without selection, which has been found to be effective in preventing the integration of foreign DNA (Iaffaldano et al., 2016; Zhang et al., 2016). Despite the fact that particle bombardment can be used to deliver a wide range of cargo, it can also cause genome damage and random DNA integrations into the plant genome, making it difficult to detect and eliminate the transgenes (Banakar et al., 2019; Liu et al., 2019). When transgenes are continuously expressed, the genome is exposed to CRISPR agents, which increases the risk of off-target mutations and chimeric mutants being generated (Fu et al., 2013; Pattanayak et al., 2013; Hashimoto et al., 2016). Furthermore, efficient species-specific expression systems, such as optimal promoters and terminators, as well as codon optimization, are required for plasmid-based CRISPR genome editing to be successful. When editing multiple targets, an efficient multiplexing system is also essential, and this is especially true for polyploid plants, where more than one gRNA may be required to knock out a single gene. The integration position of transgenes can also influence their expression (Matzke and Matzke, 1998). Furthermore, Cas protein expression based on DNA is toxic in some mammalian cell types and organisms (Morgens et al., 2017; Foster et al., 2018; Jiang et al., 2021). To avoid the problems that come with DNA delivery, particle bombardment can be a alternative method to deliver mRNA encoding Cas proteins along with the gRNA(s) into the plant system (Zhang et al., 2016). It is also possible to introduce CRISPR-associated ribonucleoproteins (RNPs) into plants that already contain the Cas protein and gRNA. Due to the fact that there is no recombinant DNA involved in this process when the gRNAs are chemically synthesised, plants edited by RNPs can be considered to be transgene free. RNPs, on the other hand, are only transiently present in plant cells and are degraded by endogenous nucleases and proteases, reducing the likelihood of off-target effects and mosaicism that can result from prolonged exposure of genomic DNA to CRISPR-based technologies (Kim et al., 2014; Kim et al., 2017; Liang et al., 2017). RNPs can be used for any organism that does not have delivery barriers, and there is no need to consider promoter compatibility or multiplexing strategies when using RNPs for any organism. Furthermore, multiple gRNAs can be used concurrently to target distinct genomic regions. If there is no crosstalk between the different types of CRISPR/Cas systems and orthogonal Cas proteins, they can be used simultaneously, allowing for multiple editing outcomes (Najm et al., 2018). It is also possible to use multiple types of CRISPR/Cas systems and orthogonal Cas proteins at the same time if there is no crosstalk between them, allowing for the achievement of multiple editing outcomes. CRISPR/Cas delivered via plasmid, on the other hand, causes cell or organism toxicity, which could be avoided by using RNP-mediated genome editing (Shin et al., 2016; Foster et al., 2018; Jiang et al., 2021). *Caenorhabditis elegans*, human cells, mice and plants all have been shown to benefit from RNP-mediated genome editing (Cho et al., 2013; Kim et al., 2014; Woo et al., 2015; Zuris et al., 2015; Foster et al., 2018; Li et al., 2020). Additionally, the *in vitro* and *in vivo* use of RNPs for screening gRNAs is well-established. Even though RNP-mediated genome editing does not require transcription or translation, it can be completed as soon as cells are transfected with the RNP construct (Kim et al., 2014). There is evidence of RNP-mediated genetic engineering in plant protoplasts, as well as RNP-edited plants (Jiang et al., 2021). Therefore, RNP-based CRISPR technology has the potential to generate transgene-free and improved germplasm that can be more easily commercialised, it still faces numerous technological constraints and challenges.

## Conclusion

It is well established that cytokinins play an important role in many aspects of plant growth and development, and their positive impact on grain yield is well documented. Significant efforts have been made over the last decade to improve yields by utilizing endogenous cytokinins. Reduced CKX expression has increased yield regardless of whether the crop is monocot or dicot. Likewise, according to Bartrina et al. (2011), the function of CKX genes in yield determination has been evolutionarily conserved and is of functional significance for all or most of the agronomically important crops (Bartrina et al., 2011). To achieve fine control, it appears necessary to identify the spatio-temporal expression patterns of CKX gene family members expressed in the shoot apical meristem (SAM) and/or during seed development. This information will aid in the identification of gene-specific, functionally associated markers for marker assisted selection (MAS) methods, as well as in the induction and/or detection of beneficial mutations using a targeting induced local lesions in genomes (TILLING) strategy. In fact, even the CRISPR technique will also require such in-depth understanding.

Despite their multifaceted role, manipulating cytokinins is challenging, due to their pleiotropic nature as well as their multigene family composition, which allows for spatio-temporal expression patterns (Jameson and Song, 2016). However, current genetic approaches (RNAi, CRISPR) are now been developed to specifically target members of the CKX gene family, which may result in increased seed yield, without any detrimental effect on the plant phenotype (Table 1). By targeting cytokinin metabolism at the genetic level, modern genome-editing tool, CRISPR open up new avenues for crop improvement. Moreover, the use of novel GE tools, allows for the simultaneous targeting of multiple genes by a single construct which vastly enhancing the scope of genome editing (Gasparis et al., 2018; Ogonowska et al., 2019). Combining rapidly evolving advancements in CRISPR/Cas tool with knowledge of IPT or CKX gene function could speed up the development of new, higher-yielding cultivars that could shape future agricultural. Whether IPT or CKX is targeted, and how the cytokinin level is altered, may be dependent on whether the crop is considered to be in a sink- or a source-limited environment. In addition, cytokinins have also been implicated in the response to both abiotic and biotic stress responses (Cortleven et al., 2019). As a result, targeting CKs will significantly enhance crop yields while also increasing tolerance to various environmental stress in a wide range of agronomically important plants.
